The article "A Deep Learning Model for Stroke Patients' Motor Function Prediction" was published in 2022. Journal: Appl Bionics Biomech.

# A Deep Learning Model for Stroke Patients' Motor Function Prediction

**DOI:** 10.1155/2022/8645165

**Published:** 2022-08-05

**Authors:** Abeer Abdulaziz AlArfaj, Hanan A. Hosni Mahmoud, Alaaeldin M. Hafez

**Affiliations:** ^1^Department of Computer Sciences, College of Computer and Information Sciences, Princess Nourah bint Abdulrahman University, P.O. Box 84428, Riyadh 11671, Saudi Arabia; ^2^Department of Information Systems, College of Computer and Information Sciences, King Saud University, Riyadh, Saudi Arabia

## Abstract

Deep learning models are effectively employed to transfer learning to adopt learning from other areas. This research utilizes several neural structures to interpret the electroencephalogram images (EEG) of brain-injured cases to plan operative imagery-computerized interface models for controlling left and right hand movements. This research proposed a model parameter tuning with less training time using transfer learning techniques. The precision of the proposed model is assessed by the aptitudes of motor imagery detection. The experiments depict that the best performance is attained with the incorporation of the proposed EEG-DenseNet and the transfer model. The prediction accuracy of the model reached 96.5% with reduced time computational cost. These high performance proves that the EEG-DenseNet model has high prospective for motor imagery brain-injured therapy systems. It also productively exhibited the effectiveness of transfer learning techniques for enhancing the accuracy of electroencephalogram brain-injured therapy models.

## 1. Introduction

The brain signal acquisition model (BSA) is a message model that can learn brain actions connected to patients' objectives and transform them into control motion. BSA models are widely utilized in therapy of brain-injured cases. EEG signals deliver a noninvasive resolution for the BSA model and are utilized in most brain signal systems. BSA systems have the following phases: signal reading, image analysis, controller apparatus, and signal forwarding [1–4]. The brain signal system paradigms using EEG are based on steady-state motor imagery control systems [5, 6]. Without muscle contraction, the imagery process comprises variations of muscle stimulated by the brain [7–11]. In the presented article, EEG signals are collected from cases with physical disabilities for brain-injured patients. Occupational therapy using motor imagery BSA models can motivate the injured motor to revive the nerves surrounding the injured brain parts and partly reinstate the cases ability.

Deep learning techniques are used for BSA systems, the EEG feature selection, prediction, and detection models [12–16]. The authors in [15] proposed a SVM model to predict two classes of motor imagery signals. The authors in [16] presented two weighted process prediction models, attaining higher accurate prediction [17]. EEG prediction using deep learning can outperform classical models on large database. Such models can designate properties without feature engineering. This marks the neural model a significant selection for handling motor imagery signals using on BSA. Recent research utilized various deep learning models to extract deep features from EEG signals. The authors in [15] proposed a convolutional neural network with an encoder with higher prediction accuracy than classical prediction models on the BSA EEG-2b dataset. Authors in [16] presented a belief deep learning prediction model using the Boltzmann model. Authors in [18] presented the envelope map of EEG signals by employing the Hilbert technique and constructed a motor imagery-based BSA prediction deep model. They employed the model to the BSA EEG-2 dataset and exhausted the most progressive prediction accuracy stated. Authors in [16] utilized a deep learning model depiction of multiple channel EEG signal to enhance the accuracy. The authors in [17] developed a novel 3D map vectors of EEG signals with a multi-CNN and the linking prediction model. Their system has accomplished high performance. In concept, deep learning attains operative EEG feature selection and better accuracy classification [18–20]. Nevertheless, because of the bad medical state and pervasiveness of brain-injured cases, the EEG capturing is hard with an effect on the structure of great-size dataset. The application of these models for motor imagery studies in brain-injured cases is restricted. Our model uses transfer learning process, which can efficiently tackle the mentioned challenges [21–25]. Transfer learning process is completed by transferring continual or switching discriminated data between cases. Features selected by transferal learning have resemblances and inheritance [26–28]. These features can be defined in a small-sized dataset and can confirm the efficiency of EEG deep CNN models [29–33].

In this research, the paper's contribution is as follows:

- Proposing a deep learning models with several extensions and parameter fine tuning using deep process
- Enhancing the accuracy of the BSA model for the recuperation of brain-injured patients, this research employs these deep model to process the EEG signals of brain-injured cases
- The presented model is to incorporate fine tuning with neural and transfer learning leading to the proposed EEG-DenseNet model to detect motor imagery settings
- This research approves the model within the cases to assess the accuracy of all other models. By evaluation the experiments of compared models, it can be proven that EEG-DenseNet outperforms other transfer learning models in all other platforms. The expected performance of our model scopes 96.5% accuracy for both left hands and right hands

The remainder of this paper is organized as follows: Section 2 presents the dataset description.  Section 3 introduces the proposed models and presents the experimental results and compare it versus other deep learning systems for motor imagery BSA system.  Section 4 depicts the proposed models extension, while Section 5 produces the conclusions and discussion.

## 2. Dataset Description

The EEG signal is captured from 100 cases (60 brain-injured patients and 40 healthy cases). The simulation utilizes 64-channel EEG reading device to gather data from brain-injured cases (EEG signals with motor imagery). Each experiment proceeds for 0.5 minutes; the details of one experiment is depicted in Figure 1. The recording begins with half the time of the motionless signal. Succeeding a prompt, EEG motor imagery signals are recorded for 6 seconds. There are prompts at the start and finish of motor imagery task. The sampling of signal reading has frequency of 960 Hz. In the gathering procedure, cases track the prompts to make imagery motions, such as hand movement. The time exhibited by the prompt is half the 0.5 minutes time line. The time for a single task is 6 seconds, and it includes a single sort of activity. The pause between successive actions is 5 seconds. The prompts for the hands movement acquirements are random. The simulation includes 50 hand motor acquisition.

These data items are recorded and labeled in a public dataset that we utilized for our experiments [15]. The statistics of the motor function data is depicted in Table 1.

### 2.1. Preprocessing Task

Preprocessing task comprises cleansing and downsizing. In this research, a 12–32 Hz low pass filter is utilized to remove noises [20], and then, the frequency rate is decreased from 960 to 60 Hz. EEG signals are usually tainted with the 40 to 60 Hz frequency with nosiness from wires and other apparatus which are seized by electrodes of the acquisition device. The signal is saved in map presentation (*N*, *M*, and *S*). *N* is defined as the count of recordings trials and is set to a constant equal to 3 which is usually enough. *M* defines the channels number; *S* defines the count of sampling items per channel. This research utilizes the brain-injured patients' EEG that has motor imagery containing hand movement. The data recorded for each case is divided into three data subsets namely: training, validation, and testing. There is a 100 trial recording for each case including motor imagery task. For each case, 90 data items are utilized for training, 15 for validation and 15 for testing. Randomly, *K* cross-validation is used where *K* = 12, to compute the expected accuracy of each case. We have 40 healthy people and 60 brain-injured patients.

### 2.2. Deep Learning Phase: The Proposed EEG-DenseNet Model

EEG-DenseNet is a dense CNN model for handling EEG signals. It is trained with small-sized dataset, and it can yield a neuro instruction.  Table 2 displays the graphical construct and the definite factors of the EEG-DenseNet deep system. The input has dimension of (*M* and *S*): *M* defines the channels number, and *S* defines the count of sampling items per channel. This research utilizes the Adam optimizer [18, 20, 21] and optimizes the entropy loss ReLu function. The proposed EEG-DenseNet is depicted in Figure 2.

### 2.3. Incorporation of Fine Tuning in the EEG-DenseNet

The efficiency of transfer learning is influenced by many parameters. One of these parameters is correspondence among the training source input and the destination signals. The greater the correspondence, the greater the fine tunings outcome. The factors attained by the initial input and CL of the EEG-DenseNet are the elementary factors (for instance, selecting a definite visual filter from the initial layers) [31–36]. The last layers select definite features (for instance, the system can recap the feature representation map distinctly and get the finest feature maps). In the simulation, the database size is rather small. To evade overfitting, the tuning of the deep learning model is done into the depicted stages:

- Adjust the factors of the output layer. Our model uses transfer learning for the initial layers, and adjust the classifier parameters
- Modify the model CL parameters to fittingly diminish the learning level and epochs count. The learning level is comparatively low because the operative system weights are utilized for model tuning. If the learning level is elevated, the system can be modified rapidly and dismisses the initial weights. After tuning, this research selects to update all parameters [37, 38]. The EEG-DenseNet model was formerly executed on large datasets, which undetectably extended the previously trained data, and its accuracy is valuable to the new dataset. Hence, fine model tuning will enhance the model to attain higher results utilizing only limited number of epochs
- Begin the training stage and compute the parameters of the transfer learning model

The proposed model utilizes both the EEG feature selection captured in the transfer learning model and fine model tuning. This creates a robust adaptive model with parameter tuning for better motor imagery recognition.

Fine tuning randomly set the weights of the pretrained network. Different datasets are utilized in the neural convolution for relearning. Also, weights are utilized on the preceding convolutional layers, and the preliminary weights on the preceding layers are set. The experiments produce better grouping of the unused layers and the fine-tuned layers, as depicted in Figure 3.

## 3. Results and the Prediction Performance

Our research uses the training, validation, and testing datasets of each case into the deep learning models under comparison along with our model.  Figure 4 displays the depiction of the expected precision of a single deep learning method. As perceived, the EEG-DenseNet method achieves the highest precision. The expected prediction precision of the EEG-DenseNet method from all cases is reaching 96.5%. The model learning parameters are depicted in Table 3. The expected total accuracy of healthy cases and brain-injured cases is depicted in Figure 2. We evaluated the statistical *t*-test of the prediction performance linking to the 100 cases using the support vector machine, latent Dirichlet allocation, and our EEG-DenseNet model, with *p* value of 5.19 × 2^−10^. It is depicted that pr is about 0.055, and the prediction precision has shown momentous variances. It implicates that enhancement of our model is higher. For the input signals, prediction accuracy of the support vector machine, latent Dirichlet allocation classifier, and our model are investigated, and the experiments are depicted in Table 4. It can be proved from the precision of our model that it outperforms other classifiers. In Figure 5: the accuracy of the EEG-DenseNet for 11 cases C1 to C11 (6 healthy: C1 to C6 and 5 brain-injured patients C7 to C11) is depicted.

We used the following definitions for the accuracy, sensitivity, and specificity:

(1) $$\begin{array}{c} \text{Accuracy}=\frac{\text{TP}+\text{TN}}{\text{TP}+\text{FP}+\text{FN}+\text{TN}}, \end{array}$$

(2) $$\begin{array}{c} \text{Sensitivity}=\frac{\text{TP}}{\text{TP}+\text{FP}}, \end{array}$$

(3) $$\begin{array}{c} \text{Specificity}=\frac{\text{TN}}{\text{TN}+\text{FN}}, \end{array}$$

where TP is the true positives, TN is the true negatives, FP is the number of false positive cases, and FN is the number false negative cases.

## 4. The Proposed Model Extension

### 4.1. Accuracy

Three extension models have been developed on the proposed EEG-DenseNet method. The starting model is to statistically set the parameter of the deep learning model; then, a different subset is fed in for model (the extension method is named EEG-DenseNet_E1).

The second extension model is to halt the variation of the weights in the block 1 of the proposed CNN in the transfer learning model and start retraining the other layers such that different weights can be attained (the processed extension model is called EEG-DenseNet_E2).

The third extension model is analogous to the second extension model, with the weights of both blocks in the proposed CNN unchanged (the processed extension model is called EEG-DenseNet_E3).

The three extension systems are compared. The expected prediction accuracies of 11 cases are depicted in Table 5. It depicts the accuracy of the various extension models. The second model has the best prediction result.

It can be depicted from Table 6 that the prediction accuracy of the EEG-DenseNet_E2 model outperforms the other two extension models. The performance results prove that model of partly unchanging parameter values is higher than the other model of the total model weight starting point. It can be depicted from Table 6 that the prediction performance from EEG-DenseNet_E2 model is higher than the results of the EEG-DenseNet_E3 model. The reason for that is that the selected features in the second one are the definite features linked to the motor imagery. By keeping the parameter values of the second block unchanged, the capability of model classification is decreased, so the accuracy is reduced.

As a final note, the experimental results realized from the EEG-DenseNet_E2 model are as shown: in the EEG-DenseNet method, it is proven that deep factors are selected in the first one, while more specified features are extracted in the second block of the CNN structure.

Performance comparison between our model and other models in terms of accuracy is depicted in Table 6.

### 4.2. Computational Complexity

In deep learning model, time complexity measurement is one of the norms for computing the model performance. The novelties of several models are established using the time computational complexity. To minimize time complexity, we substitute the multiplication operations into parallel addition operations. In this article, the research computed the floating-point operations per second (FLOPs) of all models to compute the time and space computational load of the proposed model [27].

The count of the FLOP operations controls the training time and the classification time of the proposed model. If the CPU time are getting time consuming, it can affect the model training and classification CPU time to need a high time complexity, and it is impossible to achieve the real-time requirements.

Memory requirements (MEM) are also important to compute the separability of the hardware modules of the module functionality. MEM computes the count of factors for optimizing the method. In memory restriction, the higher the number of the method parameters, the greater the quantity of input needed for model training. The size of the input in actual situations is typically not too high that deems the system modeling overfits.

In this article, floating-point operations per second and MEM of all the methods are utilized to compute the time and space computational load, as depicted in Table 7. It is shown from the mentioned table that the requirements for the EEG-DenseNet training are less than the other compared models, thus decreasing the count of operations and the parameters to fit real-time requirements. The training computation time of the EEG-DenseNet model is lower than other compared models.  Table 8 depicts the time and space requirements for the compared model classification.

In Table 9, we display the statistics for using EEG-DenseNet model with and without fine tuning depicting the correctly and incorrectly predicted cases. Also it declares the qualitative reliability Kappa metric as well as average square error. From Table 8, it is clear that incorporating fine tuning in the deep learning model will accentuate the model performance.

In Tables 10 and 11, we display the confusion matrixes for the EEG-DenseNet model with fine tuning for 100 cases for left hand and right hand.

## 5. Conclusions

In this article, the research was to determine if the proposed EEG-DenseNet model that incorporated fine parameter tuning with deep learning can be efficiently utilized for small-sized input. The presented model is primarily used for the input signals of normal cases and brain-injured cases. The simulation can prove that the total prediction results of healthy cases are higher than brain-injured cases. It is more difficult to capture EEG signals from brain-injured cases as well as very costly. Brain-injured patients have hard time staying motionless without eye blinking or involuntary movements that frequently infect the captured EEG signals. Moreover, brain damage can extremely alter the lively properties of the EEG data, thus aggregating the uncertainty of the EEG distribution. It is an important issue to attain a large size and better quality EEG signals from brain-injured cases. It should be noted that the accuracy of patients' EEG actions may not accomplish the required effect, which are prospective parameters impacting the final performance results.

This article investigated the input data of the whole cases both healthy and brain-injured patients to clarify the efficacy of the data communication of models with transfer learning. These neural structure models are motivated by image processing and feature extraction. The universal features of all cases can be learned through the initial CL model layers. Deeper more specific features are extracted from experimental training. This research can use small-sized databases by ceasing the prior layers of transfer learning and diminishes the count of model parameters that has to be maximized. This research indicates that the presented model can transfer learning for the same pattern. The experimental results depict that transfer learning should be incorporated in the paradigm of EEG processing. The EEG-DenseNet outperforms other state-of-the-art neural deep learning models in motor imagery detection. The experiments prove that we can utilize small-sized dataset for training. The learning process are efficiently done on the EEG signals of brain-injured cases via transfer learning modeling.

## Figures and Tables

**Figure 1:** Data gathering process of the simulation.

**Figure 2:** EEG-DenseNet structure.

**Figure 3:** Fine tuning of the convolutional layers.

**Figure 4:** The expected prediction performance of the compared model versus our proposed model models.

**Figure 5:** The accuracy of the EEG-DenseNet for 11 cases C1 to C11 (6 healthy: C1 to C6 and 5 brain-injured patients C7 to C11).

**Table 1:** Motricity index scores.

Motor function	Mean	Standard deviation	Minimum	Maximum
Shoulder flex	2.67	0.72	0	4
Elbow flex	2.81	0.68	0	4
Wrist extensor	0.51	0.67	0	2
Finger extensor	0.15	0.35	0	1
Finger flex	0.96	0.87	0	2
Hip flex	2.71	0.63	0	4
Knee extensor	1.71	0.73	0	3
Ankle flex	1.96	0.87	0	3
Toe flex	0.86	0.77	0	2

**Table 2:** Parameter of EEG-DenseNet: T = temporal filter, DP = depth, P = point filter. K is the count of motor imagery units.

Structure	Layer	Filters	Size	Output	Activation
1	Input: input layer			*M* × *S*	
	Reshape: first convolutional layer (CL)			1 × *M* × *S*	
	Second CL	T	(1, 64)	*T* × *M* × *S*	Linear activation function
	Normalization			T× M × S	
	Depth CL	DP × *T*	(C, 1)	(DP × *T*) × 1 × *S*	Linear activation function
	Batch sizing			(DP × *T*) × 1 × *S*	
	Nonlinear activation layer			(DP × *T*) × 1 × *S*	ReLu
	Max pooling		(1, 4)	(DP × T) ×1 × S/4	
	Dropout layer (one out of four)		Probability (pr) = 0.25 or pr = 0.5	(DP × *T*) × 1 × *S*/4	
2	Separable CL	*P*	(1, 16)	*P* × 1 × *S*/4	Linear activation function
	Batch sizing			*P* × 1 × *S*/4	
	Nonlinear activation layer			*P* × 1 × *S*/4	ReLu
	Max pooling		(1, 6)	*P* × 1 × (*S*/16)	
	Failure layer		Probability = 0.35 or probability =0.6	*P* × 1 × (*S*/32)	
	Flattening out			*P* × *S*/32	
Classifier	Dense classified fully connected	*K* × (*P* × *T*/32)	Norm = 0.25	*K*	Softmax

**Table 3:** The parameters of our model.

Model parameters	Value
Learning level	0.0002
Dropout rate	0.6
Number of epochs	200
*T*	8
*P*	12
DP	3

**Table 4:** Prediction results attained by various tuned models.

Subject	Accuracy (%)		
	Proposed model	Support vector machine	Latent Dirichlet allocation
C1	97	87	84
C2	96	87	84
C3	93	77	87
C4	97	84	87
C5	94	74	84
C6	94	77	87
C9	95	84	87
C6	96	77	77
C9	98	84	74
C10	97	87	87
C11	94	87	74
Mean	98.7	84.47	79.49
Standard deviation	±4.7	±3.8	±3.4

**Table 5:** Prediction accuracy results realized by the different extension models for both hands movements.

Case	EEG-DenseNet_E1 (%)		EEG-DenseNet_E2 (%)		EEG-DenseNet_E3 (%)	
	Left hand	Right hand	Left hand	Right hand	Left hand	Right hand
C1	87	86.5	97	96	90	93
C2	80	80	97	98	87	82
C3	77	89	87	88	80	80
C4	77	86	87	85	77	77
C5	80	80	87	88	80	84
C6	87	87	90	94	87	83
C9	87	86	90	90	87	86
C6	80	80	87	89	80	84
C9	77	85	97	88	80	85
C10	77	84.9	87	86	80	80
C11	77	86	90	97	87	86
Mean	79.09	89.09	98.7	98.8	82.29	85.7
Standard deviation	±2.3	±4.3	±3.4	±4.1	±1.9	±3.3

**Table 6:** Floating-point operations per second and training CPU time of training of all methods.

Method	Average accuracy (%)	Average sensitivity (%) (percentage of patients with a dysfunction case who predicted as positive)	Average specificity (%) (percentage of patients without a dysfunction case who predicted as negative)
EEG-DenseNet	97.6%	98.1%	97.9%
DenseNet	92.4%	93.2%	92.8%
Xception	91.4%	91.6%	92.1%
ResNet	89.7%	89.8%	88.7%
VGG16	87.4%	88.2%	88.6%

**Table 7:** Floating-point operations per second and training CPU time of training of all methods.

Method	Floating-point operations per second (millions per second)	Average minutes	Standard deviation
EEG-DenseNet	0.052	142	±8.9
DenseNet	2.479	470	±8.7
Xception	6.243	409	±10.8
ResNet	3.965	616	±12.9
VGG16	13.15	855	±14.6

**Table 8:** Floating-point operations per second and training CPU time of classification all methods.

Method	Floating-point operations per second (millions per second)	Seconds
EEG-DenseNet	0.0052	12
DenseNet	0.179	40
Xception	0.243	49
ResNet	0.765	66
VGG16	0.815	85

**Table 9:** Statistics for using EEG-DenseNet model with and without fine tuning.

	EEG-DenseNet model classifier without fine tuning	EEG-DenseNet model classifier with fine tuning
Correctly predicted	0.871	0.971
Incorrectly predicted	0.139	0.039
Qualitative reliability	0.197	0.321
Average square error	0.872	0.321

**Table 10:** Confusion matrix for the EEG-DenseNet model with fine tuning for 100 cases for left hand.

		Classified cases	
		Positive	Negative
Actual cases	Positive	50	6
	Negative	4	40

**Table 11:** Confusion matrix for the EEG-DenseNet model with fine tuning for 100 cases for right hand.

		Classified cases	
		Positive	Negative
Actual cases	Positive	53	4
	Negative	3	43

## Data Availability

Data are available upon request from the authors.
